The article "Tomographic Evaluation of the Internal Adaptation for Recent Calcium Silicate-Based Pulp Capping Materials in Primary Teeth" was published in 2021. Journal: Biomed Res Int.

# Tomographic Evaluation of the Internal Adaptation for Recent Calcium Silicate-Based Pulp Capping Materials in Primary Teeth

**DOI:** 10.1155/2021/5523145

**Published:** 2021-05-08

**Authors:** A. A. Al Tuwirqi, E. A. El Ashiry, A. Y. Alzahrani, N. Bamashmous, T. A. Bakhsh

**Affiliations:** ^1^Pediatric Dentistry Department, Faculty of Dentistry, King Abdulaziz University, P.O. Box 80209, Jeddah 215-89, Saudi Arabia; ^2^Pediatric Dentistry, Taif Dental Centre, Ministry of health, Saudi Arabia; ^3^Restorative Dentistry Department, Faculty of Dentistry, King Abdulaziz University, P.O. Box 80209, Jeddah 215-89, Saudi Arabia

## Abstract

**Objectives:**

To evaluate the internal adaptation of recent pulp capping materials (TheraCal and Biodentine) relative to MTA when used as indirect pulp capping for primary teeth.

**Materials and Methods:**

Thirty primary molars were randomly allocated into three groups, group (A) was TheraCal, group (B) was Biodentine, and MTA was the control group (C). A standardized round class-V cavity (1.5 mm diameter and 2 mm depth) was prepared using a milling machine on the buccal surface of each tooth with the pulpal floor located on the dentin. Then, pulp-capping materials were applied. Finally, all teeth were restored by composite restoration. The internal adaptation of the pulp-capping materials to the dentinal surface was investigated by microcomputed tomography (Micro-CT) to determine the internal gap volume, and by optical coherence tomography (OCT) to determine the high-intensity reflection of light from the floor.

**Results:**

Based on Micro-CT findings, TheraCal showed significantly higher internal gap volume than both MTA and Biodentine (*p* < 0.001), while MTA and Biodentine did not show a significant difference in the gap volume. Based on the OCT findings, TheraCal showed a significantly higher intensity of light reflection than both MTA and Biodentine (*p* < 0.001); however, there was no significant difference between MTA and Biodentine. Pearson's correlation test showed that there was a strong positive correlation between Micro-CT and OCT (*r* = 0.686, *N* = 30, *p* < 0.001).

**Conclusions:**

Biodentine and MTA showed a comparable result in terms of their internal adaptation on the dentinal surface of the primary teeth, and both were better than TheraCal. There is a moderate to a strong positive correlation between Micro-CT and OCT in the measurement of internal adaptation of the tested pulp capping materials. OCT can be helpful and beneficial for the clinical setting and allow dentists to screen and evaluate restorations during follow-up.

## 1. Introduction

Managing dental caries approaching the pulp is a major issue in clinical dentistry. Indirect pulp capping (IPC) treatment by preserving tooth vitality is the recommended approach for the management of deep dental caries involving vital teeth [1, 2]. Although several restorative materials offer good properties in a deep cavity, not all protect the pulpal tissues during setting or during mechanical and thermal stresses. A base or liner is usually inserted at the dentin-restoration interface to protect the pulp [3]. Materials that are composed mainly of calcium silicate are considered bioactive materials, since they induce the formation of dentin bridges by releasing their ions [4, 5]. IPC promotes dental caries recovery by using a bioactive material to isolate and seal the carious lesion and promotes the regeneration and maintenance of pulp vitality [6]. A pulp capping material should be dimensionally stable, radiopaque, and insoluble in tissue fluids. It should be able to maintain a sufficient seal and exhibit biocompatibility and bioactivity. It should also be nontoxic, nongenotoxic, noncarcinogenic, and nonresorbable. However, none of the currently available biomaterials meet all these criteria [7, 8].

MTA has been available for two decades and is widely used in clinical practice, with high success rates. MTA mainly consists of calcium oxide. Calcium oxides are present in multiple forms, such as tricalcium aluminate, dicalcium silicate, and tricalcium silicate. Its long setting time has encouraged researchers to produce new types while simultaneously utilizing MTA technology. Calcium silicate-based materials, generally referred to as MTA cement, belong to a group of materials consisting primarily of dicalcium and tricalcium silicates. However, few studies have evaluated and compared the properties of these materials against ProRoot MTA [9]. Biodentine is a recently developed fast-setting cement based on tricalcium silicate. It is formed with MTA-based cement technology, with manufacturer claims of having superior handling properties and strength [10]. Biodentine was found to have physical properties comparable to those of normal dentin. Therefore, it can be used as a substitute for dentin beneath composite restorations. It can also be used as a direct and indirect pulp capping material or for endodontic perforation repair. Biodentine also induces odontoblast differentiation from undifferentiated mesenchymal cells inside the pulp [5, 11].

TheraCal is another material that was recently introduced by utilizing MTA technology and modified by adding resin to induce polymerization controlled by light-curing systems. Gandolfi et al. found that TheraCal has a lower solubility and higher capacity to release calcium than Pro-Root MTA and calcium hydroxide in a 28-day follow-up [12]. Two studies utilized TheraCal as a direct and indirect pulp capping material and found that it has a good ability to induce reparative dentin and form a dentin bridge [13, 14]. Inconsistent outcomes were found when reviewing studies that evaluated the sealing ability of these new materials. A study that evaluated the adaptation of MTA to Biodentine found that MTA has a superior sealing ability when used as a root-end filling material [10]. In another study, both Biodentine and MTA exhibited similar performances in adaptation when used for restoration when assessed by electron microscopy [15]. In another study, Biodentine showed superior adaptation compared with MTA when examined by confocal laser scanning microscopy (CLSM) [16]. The only laboratory study comparing TheraCal's sealing ability against that of MTA and Biodentine using CLSM showed that TheraCal displayed a higher sealing ability and lesser leakage than MTA and Biodentine [17].

Microleakage and the absence of secure adaptation in the tooth-restoration interface are the main factors that affect the success and longevity of dental restorations. This might cause discoloration of the restoration, recurrence of caries, hypersensitivity, development of pulpal disease, and subsequent treatment failure [18]. Souza-Junior et al. conducted a study to evaluate marginal and internal adaptation and found that an internal gap was present in the pulp line angle of restoration [19], which would cause tooth sensitivity that may lead to bond degradation and restoration failure [20]. One of the significant objectives of tooth restoration is to protect the exposed dentin against oral flora. Therefore, the interface between the dental tissue and restoration has been an area of concern in clinical dentistry, as failure to achieve an optimal seal will cause treatment failure [21]. Interestingly, the internal gaps cannot be detected by conventional X-rays. Microcomputed tomography (Micro-CT or *μ*CT) has recently been used for evaluating the internal adaptation of restorative materials [22, 23]. This new technological advancement has led to the opportunity to perform a three-dimensional quantitative and qualitative assessment, is less time consuming, and provides more detailed outcomes by considering the entire restorative interface [23–29]. Optical coherence tomography (OCT) is a new imaging modality that is considered very promising. Many features make OCT very encouraging for clinical application [30]. These advantages include noninvasiveness, lack of radiation, ease of interpretation of both soft and hard tissues, and high spatial resolution [31–33]. Furthermore, in an *in vitro* study, OCT could visualize the internal microstructures of tissues or biomaterials without the need to cut specimens [34–36].

Few studies have addressed the internal adaptation of new pulp capping materials (TheraCal and Biodentine), and they reported a dialectical outcome [10, 37, 38]. Furthermore, no research has been performed to correlate OCT with Micro-CT for the evaluation of internal adaptation of pulp capping materials. Therefore, this study aimed to evaluate the internal adaptation of recent pulp capping materials (TheraCal, Biodentine, and MTA) as indirect pulp capping materials for primary teeth. Another aim of the present study was to compare the OCT against the Micro-CT in the evaluation of the internal adaptation for recent pulp capping materials in the primary teeth.

## 2. Materials and Methods

Ethical approval for the study protocol was obtained from the Research Ethical Committee at the Faculty of Dentistry and University Dental Hospital, King Abdulaziz University, Jeddah, Saudi Arabia (4-2-2019). This study was an *in vitro* study. The study's statistical power was calculated using statistical power analysis on the findings of both Micro-CT and OCT. The study's power to detect the groups' differences was on the ideal level for the sample size used in this study and for both Micro-CT and OCT. Thirty freshly extracted noncarious primary molars were collected. The teeth were cleaned using an ultrasonic scaler and stored in distilled water at room temperature. The teeth were randomly distributed to three groups according to the pulp capping material used (*n* = 10), group (A) for TheraCal, group (B) for Biodentine, and group (C) for MTA as control. The randomization was made using Statistical Package of Social Sciences (SPSS) program version 20.0 for Windows (Armonk, NY; IBM Corp.).

### 2.1. Specimen Preparation

Cylindrical standardized class V cavity preparations were prepared in the cervical third of each tooth on the buccal surface using a milling machine under continuous water coolant spray by one operator. Each bur was replaced after five preparations. The cavity dimensions were 1.5 mm diameter and 2 mm depth, and the cavity floor was on the dentin surface.

### 2.2. Dental Pulp Capping Materials Mixing and Application

In group A, TheraCal (Bisco, USA) was applied directly using its syringe tip inside the cavity, according to the manufacturer's instruction, and cured for 20 s. In groups B and C, the mixing of the Biodentine (Septodont Saint-Maur des-Fossés, France) and MTA (Dentsply, USA) materials was carried out following the manufacturer's instruction. Then, the pulp capping material was applied using the small tip of the amalgam carrier and condensation by using a conventional amalgam condenser. Based on the manufacturer's instructions, the TheraCal is set immediately after 20 seconds of curing with the light cure. While both Biodentine and MTA are set by hydration reaction, and both need time to set. Therefore, a wet cotton pellet was applied to cover the MTA and Biodentine, and a period was given to the materials to set before final restoration, MTA for 4 h and Biodentine for 12 min. The setting time of both materials was estimated based on a previous review study for the property of MTA and Biodentine [10, 39]. Next, all teeth were restored with the 5^th^-generation bonding agent (Adper single bond, 3M ESPE, USA) followed by Filtek Z350 XT composite restoration (3M ESPE, USA) in incremental filling technique. All restorative materials were cured with the same light-curing unit (Elipar, Curing Light 2500, 3M EPSE, USA). All specimens were subjected to thermocycling (SD Mechatronic machine, Germany) for 1000 cycles between 5°C and 55°C with a dwell time of 30 s, in order to mimic the oral condition.

### 2.3. Micro-CT Scanning and Image Analysis

The utilized Micro-CT system was Skyscan (Model 1172, Skyscan Kontich, Belgium), and the reconstruction was made using the NRecon version 1.6 software. Each specimen was mounted in a sample holder, and wax was used during Micro-CT scanning to prevent movement during the measurement. The evaluation goal was to quantify the volume of the gap and the volume of total restoration for each specimen in a cubic millimeter. The first step was to define the region of interest, which is the interface between the pulp capping materials and the dentinal surface, which was done using CT-Analyser V.1.11 software. The samples were segmented in the CT slices based on their grey-scale values. Accordingly, the total restoration volume and gap volume were measured. The gap volume was computed from the inversed segmented image of the region of interest, which is the interface between the pulp capping materials and the dentinal surface and based on density. The analysis was started using the evaluation program with a one-click operation and using all images within the area of interest.

### 2.4. OCT Scanning and Image Analysis

The utilized CP-OCT (IVS-300, Santec, Japan) system was integrated into a portable PC. The CP-OCT system was fitted with an adjustable probe that projects a high scanning rate diode laser (30 kHz) and a continuous wavelength centered about 1310 nm, with a wavelength range of 100 nm. The lateral resolution for axial resolution was about 30 *μ*m and 12 *μ*m, while the sensitivity of the device was 95 dB, and the output power of the probe was within the safety limits established by the American National Standard Institute [35, 40].

The specimen was fixed on a micrometer stage, and serial tomographic B-scan images for gap assessment at every 250 *μ*m were obtained [40]. The acquired OCT scans were transferred into an external drive and reaccessed by another PC with an image analysis software (ImageJ 1.5 m9, National Institutes of Health, USA). The images were reconstructed into a grayscale representation following a previously described protocol [40]. The cavity floor was then selected, measured, and converted to a binary image containing white and black pixels. The areas with high backscattered reflections over a white background have been converted into black pixels, representing gaps.

The gap percentage on the pulpal floor of the restoration was calculated using the equation:

(1) $$\begin{array}{c} \text{Gap percentage}=\left(\text{Gap width}/\text{width of cavity floor}\right)\times 100. \end{array}$$

### 2.5. Statistical Analysis

SPSS version 21.0 was used to analyze the collected data. The significance level for the analysis was set at *p* < 0.05; the level of confidence for this analysis was 95%. The Shapiro-Wilk test of normality was used on the findings and showed a normal distribution of the data (*p* value = 0.485). Therefore, a one-way ANOVA test was used to test the findings of both Micro-CT and OCT, followed by the least significant difference test (LSD) for multiple comparisons.

In regard to the comparison between the findings of Micro-CT and OCT, a Pearson correlation test was used. The level and strength of the correlation were measured according to Akoglu [41]. The cutoff point for the strength of the correlation was set at *r* = ±0.7 between the strong and moderate and *r* = ±0.4 between the moderate and weak correlation [41].

## 3. Results

The Micro-CT findings showed that the mean of total restoration volume (mm^3^) for groups A, B, and C were 10.893 ± 1.3, 10.888 ± 1.28, and 10.877 ± 1.28, respectively, and the *p* value within the group was equal to (*p* = 1) with no significant differences between the groups. In regard to the mean of total gap volume in (mm^3^), the value for group A was 0.207 ± 0.062, for group B was 0.021 ± 0.01, and for group C was 0.023 ± 0.015. There was a significant difference between the groups (*p* ≤ 0.001).

Micro-CT findings are presented in Table 1 and Figure 1. Representative images for each group are presented in Figure 2. The mean ratio between the total gap volume and total restoration volume was 1.903 ± 0.551, 0.2 ± 0.106, and 0.213 ± 0.147 for groups A, B, and C, respectively (*p* ≤ 0.001). The LSD test was applied to the findings to determine the differences between the groups (Table 2). The TheraCal group (A) showed a significantly (*p* ≤ 0.001) higher volume of the gap compared to both Biodentine (B) and MTA (C). Biodentine (B) and MTA (C) did not show a significant difference in respect to total gap volume (*p* = 0.927). In regard to the mean ratio between the total gap volume and total restoration volume, TheraCal group (A) showed a significantly (*p* = 0.001) higher ratio compared to both Biodentine (B) and MTA (C). While Biodentine (B) and MTA (C) did not show a significant difference in respect to the mean ratio (*p* = 0.927).

The OCT findings showed that the mean percentage of High-Intensity Reflection (HIR) of light in group A was 84.79 ± 3.17, in group B was 76.98 ± 3.14, and in group C was 76.87 ± 4.42 (*p* ≤ 0.001) the findings are shown in (Table 3 and Figure 3). The LSD test was applied to the findings to determine the differences between the groups (Table 4). TheraCal group (A) showed significantly (*p* ≤ 0.001) higher HIR compared to both Biodentine (B) and MTA (C). At the same time, Biodentine (B) and MTA (C) did not show a significant difference in HIR (*p* = 0.946). OCT scans for each group are presented in Figure 4. The mean HIR percentages at the cavity floor for the different groups.

Pearson's correlation showed that there is moderate to a strong positive correlation between Micro-CT and OCT (*r* = 0.686, *N* = 30, *p* < 0.001). Scatter plots for the findings are shown in Figure 5.

## 4. Discussion

The high success of MTA as a pulp-capping agent in previous studies makes it the gold standard as a vital pulp therapy medicament. Therefore, it was selected as a control group in this study [1, 2, 10]. Biodentine and TheraCal were selected as they were recently introduced to overcome MTA problems in terms of handling and long setting time [10]. All of these materials possess similar basic composition and nearly the same biological properties, but they differ in their set time, physical, and chemical properties.

Many methods were utilized to evaluate the sealing and resistance to the leakage of dental restorative materials. These methods include the use of dye penetration, infiltration of fluids, electrochemical technique, models for bacterial leakage, and the usage of radioisotope tracers [42]. However, these methods require slicing and destruction of the specimen to assess leakage. Another obvious limitation in this method is the subjectivity in the assessment of leakage as the dye usually causes staining of sound dentin that must be differentiated from true leakage [23, 43, 44]. Moreover, the dye penetration method is assessed either by a subjective method utilizing a predetermined scale or by a quantitative evaluation using the depth of the dye infiltration. All these tests are complex and require several preparatory steps, which increase the chance of technical errors [29, 45].

On the other hand, Micro-CT and OCT are both advanced imaging techniques that have the advantage of the nondestructive nature of assessment for the internal adaptation of dental restorative materials at a micron-scale resolution [42]. OCT and Micro-CT also have the benefit of avoidance of loss of information during optical slicing of the specimen. This means the whole floor is visible for examination without any sample destruction [42, 46]. Micro-CT and OCT permit easy detection of microgaps and defective spots inside the internal structure of the restorative material in two and three-dimensional modes (2D, 3D) [28, 44]. For this reason, we adopted this imaging technique to evaluate the internal adaptation of pulp capping agents.

MTA-based pulp capping agents can prevent microleakage, promote tissue regeneration, and provide a better seal than calcium hydroxide [1, 47]. Despite their high cost to be used for IPC, this study attempted to answer the question of which of these materials have a high adaptation on the dentin of primary teeth. Furthermore, the MTA-based pulp capping materials have high biocompatibility and bioactivity, making them very valuable in maintaining vitality in the treatment of deep caries involving vital teeth [4, 5].

This study was carried out by standardization of the teeth type, shape, and size of the cavity, type of storage medium, duration of storage, and the placement of the final restoration. All of the molars were recently extracted, cleaned, and immediately stored in distilled water. According to Lee et al., distilled water gave higher shear bond strength than other utilized storage media [48]. All of these samples were prepared by the same investigator using a milling machine to produce a standard depth and width on the buccal surface of the molar teeth. The cavity standardization was performed successfully, and this was confirmed by the measurement of Micro-CT for the total restorative volume for all the groups, which did not show any significant differences, which supports the standardization protocol that was used in this study. Each of the pulp capping materials' setting time was determined based on a previous review study for the properties of MTA and Biodentine [6]. The wet cotton pellet was also applied temporarily to ensure proper hydration during the setting's chemical reaction and optimal setting of the pulp capping materials before the restorative placement.

Analysis of the results of the current study revealed that MTA and Biodentine showed a comparable outcome regarding their internal adaptation to the dentinal surface. Although MTA showed, to some extent, better adaptation than Biodentine, they did not differ significantly. This was in agreement with Mohan et al., Brenes-Valverde et al., and Juez et al. [37, 38, 49], who found that MTA and Biodentine showed similar adaptation. The high sealing ability of MTA is probably due to the setting expansion with time, which likely leads to the closure of the gaps inside the cavity [15]. Therefore, the success of this material might be due to the inherent ability for releasing calcium hydroxide combined with the high sealing ability [1, 10]. On the other hand, the high adaptation of Biodentine might be due to its capability to form hydroxyapatite crystals, which interlock chemically with the dentinal surface by penetration inside the dentinal tubules [10].

In this study, the MTA and Biodentine findings disagreed with the results of some previous studies [15, 16, 50]. However, in some of those studies, the adaptation and sealing were tested by different procedures, e.g., when used as direct pulp capping agents or for perforation repair or apical seal. Different setting environments could contribute to different results in sealing. Malhotra and Hegde found that Biodentine was superior to MTA as an apical barrier for the root's endings [50]. However, this study utilized Dye tracer and slicing of the specimens. However, our findings disagreed with this study, possibly due to the difference in the evaluation protocol and procedure. In a study by Sulaiman et al., the authors found that Biodentine had a lower gap compared to glass ionomer and MTA [15]. The methods used in their study could contribute to their different findings compared to the current study; the preparation of the tested pulp capping agents and the slicing of specimens may increase the risk of creating iatrogenic gaps and cracks.

Regarding TheraCal, the present study revealed that it had a significantly higher internal gap at the dentinal surface when compared to MTA and Biodentine. In contrast, the only laboratory study was done to evaluate the internal adaptation of TheraCal by using confocal laser microscopy found that TheraCal had high sealing when compared to MTA and Biodentine [17]. Their findings in regard to TheraCal were in disagreement with our study. However, they agreed with our study in the findings of MTA and Biodentine as they found both materials had a comparable outcome in sealing.

The materials that were tested in this study have different compositions and application methods. The powder's hydration reaction with the liquid leads to the setting and hardening of both MTA and Biodentine [10]. While based on the manufacturer's instructions, TheraCal LC is directly applied to dentin and cured without the use of any adhesive [51]. The incorporation of resin (43%) in TheraCal without the use of any adhesive might have led to the inadequate adaptation to dentin. This was confirmed in previous studies that tested the shear bond strength of TheraCal to the dentin with and without the use of adhesive. These authors found that the bond strength of TheraCal was significantly increased by the use of adhesives (11.1 MPa) compared to no adhesive use (0.8 MPa) [52, 53]. Furthermore, in a study conducted by Camilleri et al., it was reported that there is incomplete hydration in TheraCal due to insufficient diffusion of moisture from the dentin-pulp complex inside the TheraCal [54]. The incomplete settings and inclusion of resin in TheraCal could be the cause of the low adaptation.

There was a strong correlation between the two findings from OCT and Micro-CT. This correlation was in agreement with previous studies [23, 55, 56]. The significant and strong Pearson correlation coefficient value confirms that large values of Micro-CT are associated with large OCT values. Both OCT and Micro-CT possess their own features as a method for assessment. Micro-CT is not limited by specific cavity depth for evaluation of the restoration. On the other hand, OCT has imaging depth limitations. Although OCT can show a clear image by laser penetration, it cannot be utilized in cases of a deep cavity or bulky restorations. However, this was not a problem in our experiment as the cavity depth was only 2 mm, and the reported OCT imaging depth is half to 3 mm, depending on the refractive index [57].

Moreover, the current study demonstrated that OCT produced a larger percentage number of high-intensity reflections of light compared to the volumes of the gaps produced from Micro-CT analysis. Although both findings from OCT and Micro-CT were in the same direction, full recognition of the OCT mechanism of action can help to understand this phenomenon. OCT can distinguish between the different structures that are dissimilar in composition by their difference in refractive indices and light scattering. It is well known that light is affected by changes in the refractive index. Thus, if a medium having a certain refractive index and light passes from it to another medium with a different refractive index, a part of the light will be refracted and reflected [56]. In this study, OCT was used for the detection of gaps at the interface between the pulp capping material and the surface of the dentin. Voids, which are trapped air at this interface, can cause light reflection and increase the signal obtained from OCT. A phenomenon similar to this was previously noted by using OCT for interfacial gap detection [56, 58, 59].

Up to our knowledge, this study is one of the few studies that test the internal adaptation of the three advanced calcium silicate-based pulp capping materials together when used as indirect pulp capping agents. Also, the first study used and correlated the OCT with Micro-CT in the evaluation of the internal adaptation of pulp capping materials. The results of this study indicated that OCT has great potential for direct evaluation of dental restoration when used in combination with pulp capping materials. For this reason, OCT can be beneficial in clinical settings and allow dentists to screen and evaluate restorations during follow-up. In limitation, the moistened cotton pellet was used in this study temporarily to ensure proper maturation of Biodentine and MTA before restoration. However, further research may better utilize a fast-setting liner such as resin-modified glass ionomer to cap the MTA and Biodentine instead of the moistened cotton pellet's temporary application. Also, the interpretation of these results should also consider the limitations of an *in vitro* study compared to clinical trials.

## 5. Conclusion

Biodentine and MTA have comparable outcomes in terms of internal adaptation to the dentinal surface of primary teeth, and both performed better than TheraCal. Micro-CT and OCT can assess the internal adaptation of the tested dental pulp capping materials nondestructively. However, OCT has promise for the assessment of dental restorative materials in the clinical setting.

## Figures and Tables

**Figure 1:** The mean value of total gap volume obtained by Micro-CT for the different groups. (A) TheraCal. (B) Biodentine. (C) MTA.

**Figure 2:** Representative figure obtained by Micro-CT for all groups. (a) TheraCal. (b) Biodentine. (c) MTA. The first row of the pictures is showing Micro-CT models for Group (a), the second row is showing group (b), while the third row is showing group (c). In every row, (1) picture is showing a cross-sectional 2D view for the sample. (2) 3D renderings of the sample showing the color-coded thickness of the gap within the region of interest, ranging from the thinnest structures (blue) to the thickest structures (red) according to the color bar at the bottom left. (3) 3D construction model for the restoration.

**Figure 3:** OCT mean HIR percentages at the cavity floor for the different groups. (A) TheraCal. (B) Biodentine. (C) MTA.

**Figure 4:** Representative OCT images for all tested groups. (a) TheraCal. (b) Biodentine. (c) MTA. Each B-scan is showing the composite restoration and the interface between the pulp capping material and the dentinal surface. The red arrows are pointing to the area of high-intensity reflection and microgaps.

**Figure 5:** Data plots showed a significant moderate to strong correlation (*r* = 0.68) for the findings from Micro-CT and OCT.

**Table 1:** ONE-WAY ANOVA for the Micro-CT findings.

Dependent variables	Group	*N*	Mean [mm^3^]	SD	SE	*p* value
Total restoration volume	A	10	10.893	1.302	0.411	1.000
	B	10	10.888	1.283	0.405	
	C	10	10.877	1.289	0.407	
Total gap volume	A	10	0.207	0.062	0.019	<0.001^∗^
	B	10	0.021	0.010	0.003	
	C	10	0.023	0.015	0.004	
Ratio of the total gap volume to total restoration volume	A	10	1.903	0.551	0.174	<0.001^∗^
	B	10	0.200	0.106	0.033	
	C	10	0.213	0.147	0.046	

^∗^Statistically significant *p* < 0.05. (a) TheraCal. (b) Biodentine. (c) MTA.

**Table 2:** The LSD multiple comparisons for the obtained Micro-CT results.

Dependent variable	Tested groups		Mean difference	*p* value
	Comparison			
Total gap volume	A	B	0.186	<0.001^∗^
		C	0.184	<0.001^∗^
	B	A	- 0.186	<0.001^∗^
		C	-0.001	0.932
	C	A	-0.184	<0.001^∗^
		B	0.001	0.932
Ratio of the total gap to total restorative volume	A	B	1.703	<0.001^∗^
		C	1.690	<0.001^∗^
	B	A	-1.703	<0.001^∗^
		C	-0.013	0.927
	C	A	-1.690	<0.001^∗^
		B	0.013	0.927

^∗^Statistically significant *p* < 0.05. (a) TheraCal. (b) Biodentine. (c) MTA.

**Table 3:** The ONE-WAY ANOVA for the OCT findings.

Group	N	Mean percentage of HIR	SD	SE	*p* value
A	10	84.79	3.17	1.00280	<0.001^∗^
B	10	76.98	3.14	0.99348	
C	10	76.87	4.42	1.40016	

^∗^Statistically significant *p* < 0.05. (a) TheraCal. (b) Biodentine. (c) MTA.

**Table 4:** The LSD multiple comparisons for OCT results.

Tested groups		Mean difference	*p* value
Comparison			
A	B	7.80	<0.001^∗^
	C	7.91	<0.001^∗^
B	A	-7.80	<0.001^∗^
	C	0.11	0.946
C	A	-7.91	<0.001^∗^
	B	-0.11	0.946

^∗^Statistically Significant *p* < 0.05. (a) TheraCal. (b) Biodentine. (c) MTA.

## Data Availability

Data is available upon request.
